The article "Exploration of Laser Marking Path and Algorithm Based on Intelligent Computing and Internet of Things" was published in 2022. Journal: Comput Intell Neurosci.

# Exploration of Laser Marking Path and Algorithm Based on Intelligent Computing and Internet of Things

**DOI:** 10.1155/2022/7443410

**Published:** 2022-06-24

**Authors:** Gang Lu, Yide Liu, Xue Yao, Jiachen Yang, Cheng Jia

**Affiliations:** ^1^Department of Electrical Engineering & Information Technology, Shandong University of Science and Technology, Jinan, Shandong, China; ^2^Swinburne College, Shandong University of Science and Technology, Jinan, Shandong, China

## Abstract

Nowadays, laser processing technology is being used more and more in various fields, and the requirements for laser control procedures are getting higher and higher. This paper aims to study the path generation problem of laser marking technology in order to improve the efficiency of laser marking as well as the protection of the marking material. Therefore, we creatively propose two-path generation methods, namely, sawtooth parallel and contour parallel, and design the boundary curve offset algorithm and domain partition intersection algorithm for the computer simulation of the two marking paths, respectively. Through the simulation, we discussed the efficiency and marking quality of the two path generation methods and gave the conclusion that the efficiency of the sawtooth parallel path generation method is greater than that of the contour parallel path generation method under specific parameters.

## 1. Introduction

The laser [1] is an important invention of the 20th century and has been called “the sharpest knife,” “the most accurate ruler,” and “the most unusual light.” Lasers have been increasingly used in industrial processes for a variety of machining operations such as marking, welding, drilling, cutting, heat treating, and painting. Laser marking [2] is the marking of logos, characters, symbols, and images with a laser on the product surface. It is a widely used processing method with the advantages of high processing efficiency, noncontact operation, no consumables, and low impact on product surface deformation [3] and solid marking content. The hatch tool of a laser marking machine can be used for hatch-specified 2D composite profile [4], but the setting of different hatch parameters has a great impact on the processing effect of different materials. Zigzag parallel [5] hatching and profile parallel [6] hatching are the two basic ways of marking road dynamics generation. And the design of different process processing and hatching algorithms has substantial significance on whether the operation efficiency and accuracy of laser marking machine [7] can be improved.

Nowadays, in the field of laser marking, more research lies in the combination selection and optimization of process parameters [8]. Shivakoti [9] et al. investigated the selection of optimal laser beam micromarking process parameters using the fuzzy TOPSIS [10] method in the GaN laser beam [11] marking process and concluded that small pulse frequency [12], high current, and scanning speed lead to increased mark intensity. Some people have explored this area through Bessel curves [13]. And a connected Fermat spiral area filling algorithm (CFS) [14] has also been proposed, but its study has not been deeply applied to laser marking technology and cannot be applied for complex graphics [15]. Our research aims to fill this gap in the laser marking path generation algorithm.

To fill this gap, in order to fill this gap, we explore the laser marking path generation algorithm from the perspective of improving the efficiency of laser marking path generation, combining computer graphics [16] principles with the length of the laser marking path and the time of the generation algorithm as the main factors. Firstly, we propose two-path generation methods, namely direction-parallel hatching and contour-parallel hatching. Parallel directional shaded lines, also called “zigzag” shaded lines, have paths that move along line segments parallel to the initially selected reference direction. The two marking path forms are shown in Figure 1. Based on this strategy, connected paths are obtained by connecting these parallel line segments so that they either all cross from right to left (or left to right) or alternate between left to right and right to left. In contrast, contour-parallel shading uses offset line [17, 18] segments based on boundary curves as smooth shading paths similar to boundary curves. Thus, contour-parallel shadows can be generated in a spiral fashion along a curve at a constant distance from the curve boundary. Later, the domain partition intersection algorithm and boundary curve offset algorithm are proposed for both methods and verified the feasibility and generation efficiency of both algorithms by computer simulation [19].

## 2. Method

In exploring the problem of laser marking path generation, we proposed the zigzag parallel and contour parallel [20] filling path approaches and used interpolation methods [21] to fit the original pattern at a high level to enhance the marking pattern.

Usually, the first function in an M-file is the main function, which can be followed by any number of subfunctions. The main function can be called by other functions outside that file, and the main function is called by the filename of the *M* file where the function is stored.

M files can include multiple functions, and functions other than the main function are called subfunctions. Subfunctions can only be called by the main function or by other subfunctions within that file. Each subfunction begins with a function definition statement and continues until the definition of the next function or the end of the file. The subfunctions appear in any order, but the main function must appear first.

### 2.1. Original Graph Curve Fitting

#### 2.1.1. Definition of Curve Fitting

The spline curve [22] *S*(*x*) is a segmentally defined equation. Given (*n* + 1) data points and a total of *n* intervals, the cubic spline equation satisfies the following conditions:

(A) In each segment interval [*xi*, *xi* + 1] (*i* = 0, 1,…, *n* − 1, *x* increasing), *S*_(*x*)_ = *S*_*i*(*x*)_ is a cubic polynomial
(B) The following relationship is satisfied:
  (1) $$\begin{array}{c} S_{i\left(x\right)}=y_{i}\;\left(i=0,1,\ldots ,n\right). \end{array}$$
(C) *S*(*x*), the derivative *S*′(*x*), and the second-order derivative *S*^″^(*x*) are all continuous in the interval [*a*, *b*], that is, the *S*(*x*) curve is smooth. So *n* cubic polynomial segments can be written as

(2) $$\begin{array}{c} S_{i}\left(x\right)=a_{i}+b_{i}\left(x-x_{i}\right)+c_{i}{\left(x-x_{i}\right)}^{2}+d_{i}{\left(x-x_{i}\right)}^{3}, \end{array}$$

where *i* = 0, 1,…, *n*−1, and *a*_*i*_, *b*_*i*_, *c*_*i*_, *d*_*i*_ represent the 4*n* unknown coefficients.

#### 2.1.2. Request a Solution

Interpolation and continuity:

(3) $$\begin{array}{c} S_{i}\left(x_{i}\right)=y_{i},\\ S_{i}\left(x_{i+1}\right)=y_{i+1}, \end{array}$$

where *i* = 0, 1,…, *n* − 1.

Differential continuity:

(4) $$\begin{array}{c} S_{i}^{\prime }\left(x_{i+1}\right)=S_{i+1}^{\prime \prime }\left(x_{i+1}\right),\\ \;S_{i}^{\prime \left(x_{i+1}\right)}=S_{i+1}^{\prime \prime }\left(x_{i+1}\right), \end{array}$$

where *i* = 0, 1,…, *n* − 2.

Differential equation of a spline curve:

(5) $$\begin{array}{c} S_{i}\left(x\right)=a_{i}+b_{i}\left(x-x_{i}\right)+c_{i}{\left(x-x_{i}\right)}^{2}+d_{i}{\left(x-x_{i}\right)}^{3},\\ S_{i}^{\prime \left(x\right)}=b_{i}+2c_{i}\left(x-x_{i}\right)+3d_{i}{\left(x-x_{i}\right)}^{2},\\ S_{i}^{\prime \prime }\left(x\right)=2c_{i}+6d_{i}\left(x-x_{i}\right). \end{array}$$

Bring the following step size *h* into the conditions of the spline curve:

(6) $$\begin{array}{c} h_{i}=x_{i+1}-x_{i}. \end{array}$$

Thus, we can deduce

(7) $$\begin{array}{c} a_{i}=y_{i},\\ a_{i}+h_{i}b_{i}+h_{i}^{2}c_{i}+h_{i}^{3}d_{i}=y_{i+1},\\ b_{i}+2h_{i}c_{i}+3h_{i}^{2}d_{i}-b_{i+1}=0,\\ 2c_{i}+6h_{i}d_{i}-2c_{i+1}=0. \end{array}$$

We assume that

(8) $$\begin{array}{c} m_{i}=S_{i}^{\prime \prime }\left(x_{i}\right)=2c_{i}. \end{array}$$

Thus, we can deduce the following result:

(9) $$\begin{array}{c} 2c_{i}+6h_{i}d_{i}-2c_{i+1}=0. \end{array}$$

It is equivalent to the following equation.

(10) $$\begin{array}{c} m_{i}+6h_{i}d_{i}-m_{i+1}=0. \end{array}$$

Thus, the following formula is derived as

(11) $$\begin{array}{c} d_{i}=\frac{m_{i+1}-m_{i}}{6h_{i}}. \end{array}$$

We substitute *c*_*i*_, *d*_*i*_ into

(12) $$\begin{array}{c} y_{i}+h_{i}b_{i}+h_{i}^{2}c_{i}+h_{i}^{3}d_{i}=y_{i+1}, \end{array}$$

we can derive the formula:

(13) $$\begin{array}{c} b_{i}=\frac{y_{i+1}-y_{i}}{h_{i}}-\frac{h_{i}}{2}m_{i}-\frac{h_{i}}{6}\left(m_{i+1}-m_{i}\right). \end{array}$$

From the range of values of *i*, there are (*n* − 1) equations but (*n* + 1) unknowns *m*. To solve the system of equations, two additional equations are required. So some restrictions need to be placed on the differentiation of the two endpoints *x*_0_ and *x*_*n*_. Here, we use not-a-knot [23] to solve the problem.

Specify the cubic differential matching of the spline curve.

(14) $$\begin{array}{c} S_{0}^{\prime \prime \prime }\left(x_{1}\right)=S_{1}^{\prime \prime \prime }\left(x_{1}\right),\\ S_{n-2}^{\prime \prime \prime }\left(x_{n-1}\right)=S_{n-1}^{\prime \prime \prime }\left(x_{n-1}\right). \end{array}$$

After that we can derive the following conclusions:

(15) $$\begin{array}{c} h_{1}\left(m_{1}-m_{0}\right)=h_{0}\left(m_{2}-m_{1}\right),\\ h_{n-1}\left(m_{n-1}-m_{n-2}\right)=h_{n-2}\left(m_{n}-m_{n-1}\right). \end{array}$$

The new coefficient matrix of the system of equations can be written as

(16) $$\begin{array}{c} \left[\begin{array}{cccccc} -h_{1} & h_{0}+h_{1} & -h_{0} & \cdots & \cdots & 0\\ h_{0} & 2\left(h_{0}+h_{1}\right) & h_{1} & 0 & \; & \vdots \\ 0 & h_{1} & 2\left(h_{1}+h_{2}\right) & h_{2} & 0 & \vdots \\ \vdots & 0 & \ddots & \ddots & \ddots & 0\\ 0 & \cdots & 0 & h_{n-2} & 2\left(h_{n-2}+h_{n-1}\right) & h_{n-1}\\ 0 & \cdots & \cdots & -h_{n-1} & h_{n-2}+h_{n-1} & -h_{n-2} \end{array}\right]. \end{array}$$

### 2.2. Introduction to Matlab Functions

The polyshape function [24] creates a polygon defined by two-dimensional vertices and returns an object with attributes describing its vertices, solid regions, and holes.

The polybuffer function implements the creation of a buffer around a point, line, or polyshape object. Its boundary will be input to the polyshape object buffer polyin a distance *d*. For positive values of *d*, the solid area boundary polyin expands by unit *d* and the hole boundary shrinks by unit *d*. The negative values of *d* shrink the solid boundary and expand the hole boundary.

The Intersect function is the intersection of a polyshape object. It can return the intersection of a closed curve and a line, and determine which parts of the line are inside and outside the closed curve.

### 2.3. Boundary Curve Offset Based on Contour Parallel Path

Decompose the original figure into *n* simple figures, denote the centroid [25] of each simple figure, GI represents the center point of each simple graph and the *S*_*i*_ represents the area of each simple figure, yielding the central point coordinates of the original graph as

(17) $$\begin{array}{c} x=\frac{\sum_{n}^{i=1}G_{ix}S_{i}}{\sum_{i}^{n}S_{i}},\\ y=\frac{\sum_{n}^{i=1}G_{ix}S_{i}}{\sum_{i}^{n}S_{i}}. \end{array}$$

Thus, the maximum distance from any point (*X*, *Y*) on the road strength to the center of the path is obtained as:

(18) $$\begin{array}{c} d=\max\left(\sqrt{{\left(X-x\right)}^{2}+{\left(Y-y\right)}^{2}}\right.. \end{array}$$

For the contour parallel line hatching problem, we use the buffer function polybuffer for computer simulation.

(19) $$\begin{array}{c} \text{polyout}=\text{polybuffer}\left(\text{polyin},\text{d}\right). \end{array}$$

Returns a polyshape object with a boundary that creates a buffer at distance *d* based on the input polyshape object polyin. For positive values of *d*, the solid area boundary of polyin is expanded by *d* units and the hole boundary is shrunk by *d* units. Negative values of *d* shrink the solid boundary and expand the hole boundary.

### 2.4. Domain-Distinct Intersection Algorithm for Self-Intersecting Graphs Based on Zigzag Parallel Paths

For the serrated parallel path, we propose a regionalized closed curve [26] and a straight-line intersection algorithm. Firstly the original graph is regionalized according to the concave and convex points. The original graphics and the zoning graphics are shown in Figures 2 and 3 respectively. Afterwards, using a straight line *y* = *a* from the top of the closed graph to the bottom in 1 mm steps in order to scan [27], using the intersect function to find the coordinates of the entry, and then according to the previous cycle can always find the coordinates of the intersection point of the line with the original graph each time *y* = *a*.

According to the above division, the region will be divided into many small blocks of all data points, each small block with an array to store the first (from left to right) of the intersection of the line, and then an array to store the second, because it is a sawtooth arrangement, so it must be the first from a small block to point to the second, and so on, the intersection of each small block will be the first from the small block of coordinates to point to the second coordinates.

The *X* and *Y* values of the coordinates of the intersection point, the next in each array position relationship will be the *X* and *Y* values of the coordinates of the intersection point of the next line and the intersection point of the line at the coordinates of the intersection point of that previous line and the graph. The scan intersection is shown in Figure 4.

## 3. Results

We conducted two simulation experiments on the designed contour parallel path boundary offset algorithm using Matlab software. The first simulation experiment was set to the inner shrinkage boundary distance of 1 mm and the hatch line spacing of 1 mm, and the second simulation experiment was set to the inner shrinkage boundary [28] distance of 0.1 mm and the hatch line spacing of 0.1 mm. Under these two sets of parameters, the total length of the hatching lines of the serrated parallel and contour parallel hatching curves were calculated, and the number of horizontal lines of the serrated parallel hatching and the number of circles of the contour parallel hatching were also calculated. The average running time (in ms) was calculated based on multiple runs of the hatching program, and the running time ratio of the program runs under different conditions was also calculated. The simulation results for the two parameters are shown in Figures 4 and 5, respectively.

### 3.1. Simulation of Boundary Curve Offset Algorithm Based on Contour Parallel Path

#### 3.1.1. Algorithm Analysis Results

We have performed an accurate analysis of the running time [29] of this algorithm and have derived the number of function calls and the time during the operation of the algorithm by running it several times. The results are shown in Tables 1 and 2.

#### 3.1.2. Analysis Results

According to the simulation experiment results, we counted the running time, the number of laps of the path, and the total length of the path for each simulation experiment, respectively. The results are shown in Table 3.

### 3.2. Simulation Results of Domain Partitioning Algorithm Based on Sawtooth Parallel Paths without Self-Intersecting Graphs

#### 3.2.1. Simulation Results

We generate the marking path according to the area division as follows. Figures 6to 11 show each of the five areas of the division. The final results are shown in Figures 12 and 13, respectively.

#### 3.2.2. Analysis of Domain Partitioning Intersection Algorithm Based on Sawtooth Parallel Paths

For this algorithm, we conducted two sets of simulation experiments with different parameters and performed statistical analysis on the number of calls and time of each function in the operation of the algorithm, and the following results are obtained in Tables 4 and 5, respectively.

#### 3.2.3. Zigzag Parallel Path Analysis

We statistically analyze the average running time, path length, and number of path entries of the zigzag parallel path algorithm, and the following results are obtained in Tables 6.

## 4. Discussion and Conclusion

Through the simulation solution, we can know that the average operation time of the zigzag parallel pattern filling and contour parallel pattern filling algorithms is 1 mm and 0.1 mm. After the fitting algorithm in this paper, we can get a nearly parallel straight line, while the contour pattern can be filled in parallel. The K value of the fitting function of the algorithm is close to 10, that is, under the same magnification, the zigzag algorithm can approach the previous value in time.

The algorithm in this paper can establish the length of two paths, that is, the distance that the laser sweeps through the whole closed figure, and the two paths are not very different [30].

However, the results of the simulation marking pattern can be seen, the simulation pattern based on the marking algorithm of the contour parallel path is more accurate, and the simulation pattern obtained by the marking algorithm of the sawtooth parallel path algorithm is relatively rough. Of course, this is also related to the design of our algorithm, and we believe that the accuracy of the serrated parallel path marking will be improved after the algorithm is continuously iterated and optimized.

## Figures and Tables

**Figure 1:** Graphical representation of zigzag parallel and contour parallel hatch.

**Figure 2:** Simulation graphics.

**Figure 3:** Domain zoning.

**Figure 4:** Scan for delivery.

**Figure 5:** Results of simulation experiment I.

**Figure 6:** Simulation experiment II partial enlargement.

**Figure 7:** Region 1.

**Figure 8:** Region 2.

**Figure 9:** Region 3.

**Figure 10:** Region 4.

**Figure 11:** Region 5.

**Figure 12:** Zigzag parallel experiment.

**Figure 13:** Zigzag parallel experiment II.

**Table 1:** Experiment I algorithm analysis.

Function name	Number of calls	Total time (s)	Self-use (s)
createCanvas	1	0.007	0.002
Getlnstance	1	0	0
hasBeenOpened	1	0.001	0.001
maybeShow	1	0.003	0.001
Polygon	30	0.039	0.017
doSetup	30	0.022	0.022
ToolbarController	1	0.005	0.004
Attributes	30	0.012	0.003
checkAttrs	30	0.001	0.001
checkClass	30	0.001	0.001
checkInputs	30	0.007	0.002
Axescheck	60	0.009	0.007
strcmpi (“parent”, *x*)	60	0.002	0.001
Lunkuo	1	2.221	0.089
Cla	1	0.007	0.003
converStringToCharArgs	30	0.001	0.001
generateArgumentDescriptor	30	0.004	0.004
isCharOrString	90	0	0
Gobjects	92	0.013	0.009
claNotify	1	0.001	0.001
Clo	1	0.003	0.003
hasDisplay	1	0	0
Hold	30	0.023	0.014
isFigureShowEnabled	1	0	0
isPublishingTest	1	0	0
isStringScalar	60	0.001	0.001
markFigure	30	0.005	0.005
Newplot	31	0.066	0.041
Newplotwrapper	1	0.061	0.001
Nextstyle	30	0.01	0.01

**Table 2:** Experiment II algorithm analysis.

Function name	Number of calls	Total time (s)	Self-use time (s)
createCanvas	1	0.007	0.002
Getlnstance	1	0	0
hasBeenOpened	1	0.001	0.001
maybeShow	1	0.003	0.001
Polygon	314	0.309	0.139
doSetup	314	0.177	0.17
ToolbarController	1	0.005	0.004
Attributes	314	0.042	0.009
checkAttrs	314	0.002	0.002
checkClass	314	0.008	0.008
checkInputs	314	0.023	0.01
Axescheck	628	0.057	0.048
strcmpi (“parent”, *x*)	628	0.009	0.006
Lunkuo	1	20.474	0.047
Cla	1	0.007	0.002
converStringToCharArgs	314	0.004	0.004
generateArgumentDescriptor	314	0.013	0.012
isCharOrString	942	0.002	0.002
Gobjects	942	0.077	0.059
claNotify	1	0.001	0.001
Clo	1	0.003	0.003
hasDisplay	1	0	0
Hold	314	0.181	0.112
isFigureShowEnabled	1	0	0
isPublishingTest	1	0	0
isStringScalar	628	0.003	0.003
markFigure	314	0.039	0.039
Newplot	315	0.147	0.067
newplot > ObserveAxesNextPlot	315	0.027	0.021

**Table 3:** Comparison of results of contour parallel experiments.

Experimental group	1	2	3	4	5	Average time	Number of laps	Average time ratio	Circumference
Time(s)									
Number of experiment									
1	1.937	1.952	1.995	1.959	2.103	1.989	11	10.436	896.820
2	20.583	20.534	20.51	21.169	21.002	20.759	110		10017

**Table 4:** Algorithm analysis based on zigzag parallel path simulation experiment I.

Function name	Number of calls	Total time (s)	Self-use time (s)
createCanvas	1	0.007	0.002
getlnstance	1	0	0
hasBeenOpened	1	0.001	0.001
maybeShow	1	0.003	0.001
ToolbarController	1	0.005	0.004
axescheck	6	0.002	0.002
strcmpi (“parent”, *x*)	6	0.001	0.001
c2_iuci	1	0.363	0.035
cla	1	0.006	0.002
gobjects	14	0.002	0.002
claNotify	1	0.001	0.001
clo	1	0.003	0.003
hasDisplay	1	0	0
hold	6	0.009	0.005
isFigureShowEnabled	1	0	0
isPublishingTest	1	0	0
isStringScalar	6	0	0
markFigure	6	0.002	0.002
newplot	7	0.059	0.041
newplot > ObserveAxesNextPlot	7	0.008	0.002
newplot > ObserveFigureNextPlot	7	0.001	0.001
newplotwrapper	7	0.063	0.002
area	153	0.012	0.007
intersect	51	0.034	0.028
numboundaries	408	0.011	0.01
numsides	102	0.004	0.003
perimeter	153	0.01	0.006
checkAndSimplify	51	0.204	0.166
checkArray	867	0.003	0.003
checkConsistency	408	0.001	0.001
checkinput	51	0.007	0.003
checkPointArray	51	0.003	0.003
NumHoles	102	0.002	0.002
NumRegions	102	0.003	0.003
getXY	51	0.004	0.004
isEmptyShape	408	0.014	0.002
isEqualShape	51	0.035	0.004
parselntersectUnionArgs	51	0.001	0.001
polyshape	102	0.221	0.01
settings	1	0.001	0
settings	1	0.001	0.001
usejava	1	0.001	0

**Table 5:** Algorithm analysis based on zigzag parallel path simulation experiment II.

Function name	Number of calls	Total time (s)	Self-use time (s)
createCanvas	1	0.007	0.002
getlnstance	1	0	0
hasBeenOpened	1	0.001	0.001
maybeShow	1	0.003	0.001
ToolbarController	1	0.005	0.004
axescheck	6	0.002	0.002
strcmpi (“parent”, *x*)	6	0.001	0.001
c2_iuci	1	2.476	0.08
cla	1	0.006	0.002
gobjects	14	0.002	0.002
claNotify	1	0.001	0.001
clo	1	0.003	0.003
hasDisplay	1	0	0
hold	6	0.009	0.005
isFigureShowEnabled	1	0	0
isPublishingTest	1	0.001	0.001
isStringScalar	6	0	0
markFigure	6	0.002	0.002
newplot	7	0.057	0.038
newplot > ObserveAxesNextPlot	7	0.008	0.002
newplot > ObserveFigureNextPlot	7	0.001	0.001
newplotwrapper	7	0.061	0.002
area	1593	0.103	0.048
intersect	531	0.283	0.251
numboundaries	4248	0.099	0.085
numsides	1062	0.026	0.021
perimeter	1593	0.092	0.044
checkAndSimplify	531	1.945	1.653
checkArray	9027	0.029	0.029
checkConsistency	4248	0.01	0.01
checkinput	531	0.023	0.011
checkPointArray	531	0.01	0.01
NumHoles	1062	0.012	0.012
NumRegions	1062	0.023	0.023
getXY	531	0.012	0.012
isEmptyShape	4248	0.119	0.021
isEqualShape	531	0.272	0.016
parselntersectUnionArgs	531	0.004	0.004
polyshape	1062	2.043	0.075
settings	1	0.001	0
settings	1	0.001	0.001
usejava	1	0.001	0

**Table 6:** Analysis of each factor of the zigzag path simulation experiment.

Experimental group	1	2	3	4	5	Average time	Average time ratio	Circumference	Number of articles
Time									
Number of experiment									
1	0.073	0.076	0.076	0.074	0.078	0.0754	1.0026	9176	957
2	0.075	0.075	0.075	0.076	0.077	0.0756		868	85

## Data Availability

The datasets for this study can be found in the (official website of APMCM) (https://www.apmcm.org/detail/2403).
